# Construction of a Nomogram Model for Predicting Pleural Effusion Secondary to Severe Acute Pancreatitis

**DOI:** 10.1155/2022/4199209

**Published:** 2022-03-19

**Authors:** Bing-Mei Zhou, Zhao-Lei Qiu, Kai-Xuan Niu, Yin-E. Wang, Fu-Chen Jie

**Affiliations:** Department of Emergency, The First Affiliated Hospital of Bengbu Medical College, Bengbu 233000, Anhui, China

## Abstract

**Background:**

This study aims to investigate the risk factors of pleural effusion (PE) secondary to severe acute pancreatitis (SAP) and to build a nomogram model.

**Methods:**

The clinical parameters of SAP patients admitted to the emergency department of the First Affiliated Hospital of Bengbu Medical College from January 2019 to August 2021 were retrospectively collected. The independence risk factors of PE secondary to SAP were analyzed by univariate analysis and multivariate logistic regression analysis. A nomogram risk prediction model was established and validated through the area under the ROC curve.

**Result:**

Two hundred twenty-two SAP patients were included for analysis, of which 65 patients experienced secondary PE. The incidence of PE secondary to SAP was 29.28% (65/222). Logistic regression analysis showed that serum albumin (ALB) (OR = 0.830, 95% CI: 0.736∼0.936), fibrinogen (FIB) (OR = 4.573, 95% CI: 1.795∼11.648), C-reactive protein (CRP) (OR = 1.046, 95% CI: 1.009∼1.083), acute physiology, chronic health score system (APACHE-II) score (OR = 1.484, 95% CI: 1.106∼1.990), and sequential organ failure score (SOFA) (OR = 43.038, 95% CI: 2.030∼4.548) were independent risk factors for PE secondary to SAP (*P* < 0.05) and entered into the nomogram. The nomogram showed robust discrimination with an index of concordance of 0.755 and an area under the receiver operating characteristic curve of 0.837 (95% CI: 0.779∼0.894).

**Conclusion:**

We developed a nomogram model for PE secondary to SAP with ALB, FIB, CRP, APACHE-II scores, and SOFA scores. The nomogram model showed good discrimination and consistency, and it can better predict the risk of PE secondary to SAP.

## 1. Introduction

Severe acute pancreatitis (SAP) is the most serious type of acute pancreatitis (AP) with persistent (>48 h) organ failure, accounting for 5%∼10% of all AP diagnoses [1]. It has the common clinical characteristics of rapid progression and a high mortality rate of 36%∼50% [2]. Pleural effusion (PE) is one of the common complications of a wide variety of diseases, including SAP. In patients with SAP, the occurrence of PE is the pathological accumulation of fluid between layers of pleural by reason of transdiaphragmatic lymphatic blockage or pleural fistula [3]. The previous study reported that the occurrence of PE is closely related to the severity of SAP and can be used as one of the effective indicators for early prediction of the prognosis in SAP [4]. Prediction of early onset of PE for patients with SAP and early intervention can help to improve their prognosis.

However, so far, the clinical diagnosis of PE secondary to SAP is still mainly based on CT, X-ray, and other imaging methods. For PE, imaging methods can help diagnose when it occurred and cannot predict its occurrence and screen high-risk patients. Therefore, it is vital to seek a simple way to screen high-risk patients for predicting PE secondary to SAP via constructing a risk prediction model and formulating prevention and control action plans. In the SAP process, inflammation in the pancreas could lead to an inflammatory response syndrome [5]. Also, previous research reported that Acute Physiology and Chronic Health Evaluation (APACHE-II) and Sequential Organ Failure Assessment (SOFA) are closely related to the severity of SAP [6, 7]. In this study, we retrospectively analyzed the general data and clinical characteristics of patients with SAP who contained inflammatory indicators, APACHE-II score, and SOFA score, screened out independent risk factors for PE secondary to SAP, and constructed a nomogram prediction model based on these factors. The risk prediction model will provide supporting evidence to achieve the purpose of early diagnosis and early intervention.

## 2. Materials and Methods

### 2.1. Study Subjects

The general data and clinical characteristics of patients with SAP admitted to the emergency department of the First Affiliated Hospital of Bengbu Medical College from January 2019 to August 2021 were retrospectively collected. Patients eligible for the analysis need to comply with the following inclusion and exclusion criteria. The inclusion criteria were as follows: (1) patients diagnosed with SAP using the Guidelines for Diagnosis and Treatment of Acute Pancreatitis in China (2019) [8]; (2) patients with complete data from chest examination; (3) patients admitted within 72 hours; (4) patients without a severe postheart failure, liver damage, or renal dysfunction; (5) patients without serious infection recent; and (6) patients have not received treatment of anti-inflammatory or inhibited pancreatic enzyme secretion. The exclusion criteria were as follows: (1) patients with acute exacerbation of chronic pancreatitis; (2) patients accompanied by malignant tumors or diseases of the hematopoietic system; (3) patients accompanied by rheumatic immune or endocrine diseases; and (4) patients with incomplete data. This study protocol was approved by the Ethics Committee of the First Affiliated Hospital of Bengbu Medical College (number: 2020KY073).

### 2.2. Study Design

Two hundred twenty-two patients were divided into PE secondary to SAP (PE) and control groups according to whether PE complications occurred. We reviewed medical records and collected general data and clinical parameters of patients with SAP. The general data of SAP patients included age, body mass index (BMI), gender, past medical history of fatty liver, hyperlipidemia and cholecystitis, smoking history, alcoholic drinking history, APACHE-II score, and SOFA score. The clinical parameters of SAP patients included white blood cell (WBC), neutrophil count (NEU), ALB, calcium (Ca), FIB, fasting blood plasma glucose (FPG), C-reactive protein (CRP), amylase (AMY), and lipase (LIP). The abovementioned lab test results of SAP patients were evaluated in the first test after admission. The APACHE II score consists of three parts: 12 acute physiology variables, age, and chronic health status. The theoretical score is 0 to 71 points; a higher score indicates more severe illness. The SOFA scores were determined by the function of the respiratory, coagulatory, liver, cardiovascular, kidney, and nervous systems, each scored from 0 to 4. The higher the score, the more severe the organ failure and the worse the prognosis. The primary endpoint of our study was whether the patient developed PE complications during hospitalization. The diagnosis was mainly based on imaging examinations (X-ray, CT, and B-ultrasound).

### 2.3. Statistical Analysis

Sciences SPSS software version 23.0 was used to perform statistical analysis. Normal distributed quantitative variables were expressed as ‾*x* ± *s*; otherwise, they were described as the median and interquartile range. The qualitative data were expressed as a rate (%) and analyzed using the *χ*^2^ test. Univariate analysis and multivariate logistic regression analysis were performed on the general data and lab test results of SAP patients to analyze the independent risk factors of PE secondary to SAP. The R software RMS package was used to construct a nomogram model predicting PE secondary to SAP, validated using the bootstrap self-sampling method. The C-index was used to determine the model distinction, and the area under the ROC curve evaluates the model's predictive power. The difference was statistically significant with a *P* value of <0.05.

## 3. Results

### 3.1. Univariate Analysis of Risk Factors for PE Secondary to SAP

Two hundred twenty-two SAP patients were included for analysis, of which 65 patients experienced secondary PE. The incidence of PE secondary to SAP was 29.28% (65/222). Compared with the control group, patients with PE secondary to SAP had higher WBC, NEU, FIB, CRP, APACHE-II, and SOFA scores, and lower levels of ALB, GLU, and AMY (all *P* < 0.05) (Table 1).

### 3.2. Multivariate Analysis of Risk Factors for PE Secondary to SAP

The results showed higher FIB (OR = 4.573, 95% CI: 1.795∼11.648), CRP (OR = 1.046, 95% CI: 1.009∼1.083), APACHE-II (OR = 1.484, 95% CI: 1.106∼1.990), and SOFA (OR = 43.038, 95% CI: 2.030∼4.548) scores, and lower ALB (OR = 0.830, 95% CI: 0.736∼0.936) were related to PE secondary to SAP (Table 2).

### 3.3. Development of PE Secondary to SAP-Predicting Nomogram

A nomogram incorporating ALB, FIB, CRP, APACHE-II, and SOFA scores was developed and presented as shown in Figure 1. For one patient, the corresponding points of ALB, FIB, CRP, APACHE-II, and SOFA scores are 29, 58, 24, 27, and 98, respectively. The sum of the points is located on the total points axis and corresponds to the probability shown further (risk of PE secondary to SAP).

### 3.4. Evaluation of the Nomogram Model

The bootstrap method was used to resample 1000 times to evaluate the developed nomogram model. The calculated C-index value is 0.716, which indicates that the prediction model has good discrimination. The AUC for the developed nomogram model is 0.773 (95% CI: 0.712∼0.844), which has a high predictive value (Figure 2).

## 4. Discussion

PE is one of the common complications of SAP, which also acts as a vital sign of systemic inflammation in AP. It is closely related to the progression and prognosis of SAP. Once it occurs, the patient's condition deteriorates rapidly, and the incidence of various complications and mortality is significantly increased [9]. Previous research has reported that the incidence of PE in non-mild AP patients has increased significantly that could predict the progression of AP, with an AUC of 0.622 [10]. The incidences of PE in AP and SAP were 42.02% and 72.82%, with significant differences [11]. Other studies have found the incidence of AP complicated with PE to be 11.26% and 39.80%, and the fluid volume of pleural effusion was related to the severity of AP [12,13]. In our study, the incidence of PE secondary to SAP was 29.28% (65/222), which was slightly lower than related reports at home and abroad but still at a high level.

PE secondary to SAP is mainly due to transdiaphragmatic lymphatic blockage or pleural fistula [3,14]. The occurrence of PE is the main reason for the poor prognosis of SAP patients. Early prediction of PE and early intervention may help to improve the prognosis of patients. The key is to accurately identify risk factors for SAP complicated with PE and construct an individualized predictive model. This study retrospectively analyzed the general data and clinical parameters of SAP patients in the past three years. The results showed that ALB, FIB, CRP, APACHE-II, and SOFA scores are the influencing factors of SAP complicated with PE. An elevated CRP level is one of the acute reactions of the body to infection and tissue damage, which is correlated positively with the severity of pancreatitis. Zuo L summarized AP complication with PE and its prognostic factors, and the results showed that CRP (OR = 1.656, 95% CI: 1.379∼1.992, *P* < 0.001) is an independent risk factor for AP complication with PE [11]. It may be because of the significant increase of basal metabolic rate in SAP patients under stress and the release of various systemic inflammatory mediators such as inflammatory transmitters and cytokines, leading to a rapid increase in CRP levels [5]. However, the mechanism between elevated levels of CRP and the occurrence of PE still needs further study. In addition, the release of inflammatory mediators will lead to damage of vascular endothelial cells and an increase in vascular permeability, which will promote the leakage of ALB from intravascular space to the interstitial space [9]. The capillary endothelial cell damage could also activate the internal and external coagulation systems, leading to coagulation/fibrinolysis system dysfunction, thus increasing the level of FIB [15].

The APACHE-II score is the primary tool used to evaluate the severity of pancreatitis. It can reflect the overall physiological changes of the body and has good sensitivity and specificity. The previous study has shown that the APACHE-II score is closely related to the prognosis of SAP patients and is positively correlated with mortality [16]. In addition, the APACHE-II score is also associated with inflammation indicators such as CRP and the grade of peripancreatic effusion secondary to SAP [17]. This study found that the APACHE-II score of PE secondary to SAP was 1.484 times that of the control (95% CI: 1.106∼1.990), indicating that the APACHE-II score is an independent predictor of SAP with PE.

Compared with the APACHE-II score, the SOFA score includes six organ systems such as breathing, blood, liver, cardiovascular, nerve, and kidney, which can dynamically reflect the functional status of the body's various organ systems. A higher SOFA score indicates more severe organ failure. The previous study has found that the SOFA score can predict the trend in critically ill patients' conditions and has a high value in the dynamic assessment of prognostic risk [18]. Zhou HJ [19] found that the severity of AP elevated with the increase of SOFA. In this study, the OR value of the SOFA score predicting PE secondary to SAP was 3.038, which is significantly higher than the APACHE-II score, suggesting that the SOFA score has a higher predictive value for PE secondary to SAP than the APACHE-II score.

It should be pointed out that this study has the following limitations: (1) first, this study is susceptive to selection bias because it is a single-center retrospective study with a limited sample size, which might affect the prediction accuracy. Thus, future large-scale prospective studies in multicenters should carry out a large-scale prospective study in multicenters. (2) Next, in this study, the nomogram model for predicting pleural effusion secondary to severe acute pancreatitis has not undergone external validation. (3) Finally, the therapy-related factors were not considered in this prediction model system.

In summary, we developed a nomogram model for PE secondary to SAP with ALB, FIB, CRP, APACHE-II scores, and SOFA scores. The nomogram model showed good discrimination and consistency, and it can better predict the risk of PE secondary to SAP.

## Figures and Tables

**Figure 1:** The developed nomogram of PE secondary to SAP risk.

**Figure 2:** ROC curve of the developed nomogram model for predicting the PE secondary to SAP.

**Table 1:** Univariate analysis of risk factors for PE secondary to SAP.

Indexes	Control ( = 157)	PE secondary to SAP (*n* = 65)	*t*/*x*^2^	*P*
Age	50.59 ± 18.63	51.54 ± 18.16	0.348	0.728
BMI	22.66 ± 1.45	22.68 ± 1.02	0.089	0.929
*Gender*				
Male	96 (61.15)	38 (58.46)	0.139	0.710
Female	61 (38.85)	27 (41.54)		
Fatty liver (*n* (%))	47 (29.94)	24 (36.92)	1.032	0.310
Hyperlipidemia (*n* (%))	22 (14.01)	5 (7.69)	1.719	0.190
Cholecystitis (*n* (%))	28 (17.83)	12 (18.46)	0.012	0.912
Smoking (*n* (%))	25 (15.92)	12 (18.46)	0.213	0.644
Alcohol (*n* (%))	15 (9.55)	12 (18.46)	3.141	0.065
WBC (×10^9^/L)	14.02 ± 4.11	15.45 ± 4.88	2.225	0.027
NEU	80.88 ± 8.75	84.86 ± 11.48	2.801	0.006
ALB (g/L)	38.98 ± 5.52	34.24 ± 5.96	5.680	<0.001
FIB (mg/dl)	5.33 ± 0.89	6.05 ± 0.90	5.432	0.013
GLU (mmol/L)	7.61 ± 2.78	6.82 ± 0.98	2.254	<0.001
CRP (mg/L)	102.73 ± 22.36	113.64 ± 19.46	3.431	0.025
AMY (U/L)	173.16 ± 20.39	169.11 ± 17.46	1.401	0.001
LIP (U/L)	1232.34 ± 371.89	993.12 ± 83.94	5.126	0.163
APACHE-II score	20.47 ± 2.74	22.03 ± 2.21	4.072	<0.001
SOFA score	4.87 ± 1.31	9.58 ± 3.61	14.279	<0.001

**Table 2:** Multivariate analysis of risk factors for PE secondary to SAP.

Index	B	SE	Wald	*P*	OR (95% CI)
Age	−0.028	0.021	1.779	0.182	0.973 (0.934∼1.013)
BMI	−0.109	0.245	0.198	0.656	0.897 (0.554∼1.450)
Gender	0.888	0.736	1.456	0.228	2.431 (0.574∼10.284)
Fatty liver (*n* (%))	−1.512	0.863	3.074	0.080	0.220 (0.041∼1.195)
Hyperlipidemia (*n* (%))	1.652	1.562	1.119	0.290	5.218 (0.244∼111.394)
Cholecystitis (*n* (%))	−0.167	1.018	0.027	0.870	0.846 (0.115∼6.220)
Smoking (n (%))	0.284	0.966	0.086	0.769	1.328 (0.200∼8.813)
Alcohol (*n* (%))	0.542	1.339	0.164	0.686	1.720 (0.125∼23.740)
WBC (×10^9^/L)	0.036	0.076	0.226	0.634	1.037 (0.894∼1.203)
NEU	0.054	0.041	1.774	0.183	1.056 (0.975∼1.143)
ALB (g/L)	−0.187	0.061	9.260	0.002	0.830 (0.736∼0.936)
FIB (mg/dl)	1.520	0.477	10.154	0.001	4.573 (1.795∼11.648)
GLU (mmol/L)	−0.137	0.181	0.575	0.448	0.872 (0.612∼1.243)
CRP (mg/L)	0.045	0.018	6.114	0.013	1.046 (1.009∼1.083)
AMY (U/L)	−0.008	0.019	0.187	0.666	0.992 (0.957∼1.029)
LIP (U/L)	0.394	0.150	6.931	0.008	1.484 ( 1.106∼1.990)
APACHE-II score	1.111	0.206	29.160	0.000	3.038 (2.030∼4.548)
SOFA score	0.904	0.128	49.535	0.000	2.472 (1.920∼3.177)
Constant	−23.564	9.701	5.900	0.015	0.000

## Data Availability

All the data generated or analyzed during this study are included within this article. The processed data are available from the corresponding author upon reasonable request.

## References

[1] Lee P. J., Papachristou G. I. (2020). Management of severe acute pancreatitis. *Current Treatment Options in Gastroenterology*.

[2] Dhannoon A., Knightly N., College R. (2020). AB166. acute pancreatitis: a retrospective 5-year review of aetiology. *Epidemiology and Management*.

[3] Yang J., Zheng S., Zhang F. (2017). Correlation of disease severity with pleural effusion in patients with acute pancreatitis. *Progress in Modern Biomedicine*.

[4] Datta I. K., Haque M. (2018). Incidence and predictive value of ascites and pleural effusion for severity in acute pancreatitis. *Acute Biliary Pancreatitis*.

[5] Fukushi K., Tominaga K., Takenaka K. (2019). Severe acute pancreatitis with inflammation extending to the scrotum. *Clinical Case Reports*.

[6] Wan J., Shu W., He W. (2019). Serum creatinine level and APACHE-II score within 24 h of admission are effective for predicting persistent organ failure in acute pancreatitis. *Gastroenterology Research and Practice*.

[7] Tee Y.-S., Fang H.-Y., Kuo I.-M., Lin Y.-S., Huang S.-F., Yu M.-C. (2018). Serial evaluation of the SOFA score is reliable for predicting mortality in acute severe pancreatitis. *Medicine*.

[8] Chinese Medical Association (2019). Chinese medical association journal, Chinese medical association gastroenterology branch, etc. Primary diagnosis and treatment guidelines for acute pancreatitis (2019). *Chinese Journal of General Practitioners*.

[9] Ye C., Xu Y., Wang L. (2019). Analysis of early risk factors for pleural effusion in patients with acute pancreatitis. *Hebei Medicine*.

[10] Ming G., Xiang H., He L. (2015). Evaluation value of serum Ghrelin and pleural effusion in patients with acute pancreatitis. *Chongqing Medicine*.

[11] Zuo L., Zhang H., Chen J. (2019). Factors influencing acute pancreatitis complicated with pleural effusion. *Chinese General Practice*.

[12] Zeng Q. X., Jiang K. L., Wu Z. H. (2021). Pleural effusion is associated with severe renal dysfunction in patients with acute pancreatitis. *Medical Science Monitor*.

[13] Peng R., Zhang L., Zhang Z.-M., Wang Z.-Q., Liu G.-Y., Zhang X.-M. (2020). Chest computed tomography semi-quantitative pleural effusion and pulmonary consolidation are early predictors of acute pancreatitis severity. *Quantitative Imaging in Medicine and Surgery*.

[14] Lam S., Banim P. (2014). Massive loculated pleural effusion in a patient with pancreatic pseudocyst due to alcohol-related chronic pancreatitis. *BMJ Case Rep*.

[15] Wang L.-X., Gao J.-L., Wu G.-K., Tian X.-H., Gao W. (2013). Risk factors and nursing strategies for severe acute pancreatitis complicated with multiple organ dysfunction syndrome. *World Chinese Journal of Digestology*.

[16] Alam M., Agrawal P., Singh R. K., Singh K. K., Pratap D. (2021). Comparative assessment of severity and prognosis of acute pancreatitis through APACHE II and HAPS predictor models. *International Journal of Research in Medical Sciences*.

[17] Harshit Kumar A., Singh Griwan M. (2018). A comparison of APACHE II, BISAP, Ranson’s score and modified CTSI in predicting the severity of acute pancreatitis based on the 2012 revised Atlanta Classification. *Gastroenterology Report*.

[18] Shi L., Zhang D., Zhang J. (2020). Albumin-bilirubin score is associated with in-hospital mortality in critically ill patients with acute pancreatitis. *European Journal of Gastroenterology and Hepatology*.

[19] Zhou H. J., Xue M., He X. H. (2019). Severity stratification and prognostic prediction of patients with acute pancreatitis at early phase: a retrospective study. *Medicine*.

